# Indicators of Acute and Persistent Renal Damage in Adult Thrombotic Microangiopathy

**DOI:** 10.1371/journal.pone.0030886

**Published:** 2012-01-23

**Authors:** Firuseh Dierkes, Nikolaos Andriopoulos, Christoph Sucker, Kathrin Kuhr, Markus Hollenbeck, Gerd R. Hetzel, Volker Burst, Sven Teschner, Lars C. Rump, Thomas Benzing, Bernd Grabensee, Christine E. Kurschat

**Affiliations:** 1 Department of Nephrology, Medical Faculty, Heinrich-Heine-University, Düsseldorf, Germany; 2 Renal Division, Department of Medicine and Center for Molecular Medicine, University of Cologne, Cologne, Germany; 3 Department of Hemostasis and Transfusion Medicine, Heinrich-Heine-University Medical Center, Düsseldorf, Germany; 4 Institute of Medical Statistics, Informatics and Epidemiology, University of Cologne, Cologne, Germany; 5 Department of Nephrology and Rheumatology, Knappschaftskrankenhaus, Bottrop, Germany; 6 Cologne Excellence Cluster on Cellular Stress Responses in Aging-Associated Diseases, University of Cologne, Cologne, Germany; National Cancer Institute, United States of America

## Abstract

**Background:**

Thrombotic microangiopathies (TMA) in adults such as thrombotic thrombocytopenic purpura (TTP) and hemolytic uremic syndrome (HUS) are life-threatening disorders if untreated. Clinical presentation is highly variable and prognostic factors for clinical course and outcome are not well established.

**Methods:**

We performed a retrospective observational study of 62 patients with TMA, 22 males and 40 females aged 16 to 76 years, treated with plasma exchange at one center to identify clinical risk factors for the development of renal insufficiency.

**Results:**

On admission, 39 of 62 patients (63%) had acute renal failure (ARF) with 32 patients (52%) requiring dialysis treatment. High systolic arterial pressure (SAP, p = 0.009) or mean arterial pressure (MAP, p = 0.027) on admission was associated with acute renal failure. Patients with SAP>140 mmHg on admission had a sevenfold increased risk of severe kidney disease (OR 7.464, CI 2.097–26.565). MAP>100 mmHg indicated a fourfold increased risk for acute renal failure (OR 4.261, CI 1.400–12.972). High SAP, diastolic arterial pressure (DAP), and MAP on admission were also independent risk factors for persistent renal insufficiency with the strongest correlation for high MAP. Moreover, a high C-reactive protein (CRP) level on admission correlated with renal failure in the course of the disease (p = 0.003). At discharge, renal function in 11 of 39 patients (28%) had fully recovered, 14 patients (23%) remained on dialysis, and 14 patients (23%) had non-dialysis-dependent chronic kidney disease. Seven patients (11%) died. We identified an older age as risk factor for death.

**Conclusions:**

High blood pressure as well as high CRP serum levels on admission are associated with renal insufficiency in TMA. High blood pressure on admission is also a strong predictor of sustained renal insufficiency. Thus, adult TMA patients with high blood pressure may require special attention to prevent persistent renal failure.

## Introduction

Thrombotic microangiopathies (TMA) such as HUS or TTP are rare microangiopathic thrombotic disorders characterized by hyaline thrombi in the arterial microvasculature, Coombs-negative hemolytic anemia, and thrombocytopenia. Prior to the introduction of plasma infusion and plasma exchange therapy, TMA was associated with a mortality rate of more than 90% in adults [1], [2]. In recent years, with the advent of plasma exchange in TMA mortality rate could be drastically decreased, but TMA can still be viewed as a life-threatening disorder with the outcome depending on the underlying disease, the age of the patient, severity of organ damage (e.g. kidney, heart, brain), and on the time lapse between the onset of symptoms and initiation of plasma therapy.

A variety of possible triggers such as gastrointestinal infection with *E.coli O157:H7*, *E.coli O104:H4* or *Shigella* for typical HUS and genitourinary or respiratory infections, human immunodeficiency virus infection, hormonal dysbalance, drugs, tumours, inherited and acquired defects in complement components and autoimmune diseases for TTP and adult atypical HUS have been identified [3], [4], [5]. However, in up to 30% of cases the underlying cause remains unclear. Recently, a large outbreak of *E.coli O104:H4* in Germany demonstrated the clinical severity of this disease [6]. New pathophysiological approaches identified a low activity of ADAMTS13, a metalloprotease responsible for cleavage of unusually large *von Willebrand factor* (ULvWF) multimers, to be responsible for TTP development [3], [7], [8]. However, according to epidemiologic studies ADAMTS13 activity was reduced below 5% in only 15% of patients with TMA [9], suggesting the presence of additional unrecognized risk factors predisposing for the onset and clinical course of TMA. Patients with atypical HUS may have a deficiency of complement factor H or auto-antibodies directed against this protein. Furthermore, mutations in the membrane cofactor protein gene (MCP/CD46), in the complement factor I gene, in the complement factor B gene or in the thrombomodulin gene may also be present [10], [11], [12]. In atypical HUS and selected Shiga-toxin-induced HUS cases the humanized monoclonal anti-C5 antibody eculizumab was reported to be beneficial [13], [14], [15]. In contrast to HUS patients, classic TTP patients usually present with predominant neurological symptoms. Since there is considerable clinical overlap between these two entities the disease is often referred to as HUS/TTP [16].

Presently, there is a need for risk stratification to guide therapy and follow-up. Therefore, we analysed 62 consecutive adult patients with TMA admitted to our hospital between 1989 and 2006.

## Methods

### Study design

The aim of this study was to identify clinical risk factors for acute renal failure, persistent renal insufficiency and for mortality in adult TMA patients. Data of 62 patients (22 males, 40 females) consecutively admitted to our hospital between June 1989 and June 2006 at the age of 16 to 76 years with their first episode of acute TMA were analyzed. This study was reviewed and approved by the Institutional Review Board of Düsseldorf University as exempt research without requirement for informed consent as this was review of existing data. TMA was diagnosed on the basis of clinical criteria: thrombocytopenia of less than 100,000/µl, Coombs-negative hemolytic anemia (Hb<12 g/dl, LDH>240 U/l), and the presence of more than two schistocytes per visual field in the peripheral blood smear. Other causes of severe thrombocytopenia, in particular disseminated intravascular coagulation or idiopathic thrombocytopenic purpura, were excluded. Almost all patients in this study were treated with plasmapheresis. 57 of the patients underwent plasma exchange therapy within 12 hours after admission; three patients received plasma infusion due to less severe disease. Two patients died from severe cerebral hemorrhage before initiation of plasma therapy. Medical records of all patients were examined for clinical signs of TMA and potential risk factors for the disease. In this study, we did not classify patients into TTP, HUS, or overlap syndromes by determining ADAMTS13 levels, factor H, B, I, MCP or thrombomodulin gene mutations [11], [12], [17] because these data were only available in a subset of patients. Furthermore, although the concept of ADAMTS13 deficiency or mutations in complement factors being responsible for the development of TMA is important, TMA patients still represent a very heterogenous group. Thus, the known pathophysiologic approaches are applicable to some, but not all TMA patients [9], [12], [18], [19], [20].

Clinical parameters (age, sex, SAP, DAP, MAP, white blood cell count, hemoglobin concentration, platelet count, LDH, serum creatinine, blood urea nitrogen (BUN), CRP) were analysed on admission and at discharge. For plasmapheresis, we routinely administered 250 mg methylprednisolone i.v. per day initially for the first three days followed by 1–4 mg/kg body weight of prednisone orally per day, usually at the same time as plasma therapy.

Acute renal failure (ARF) in patients with no prior history of kidney disease was defined by an increase of serum creatinine levels of >0.5 mg/dl in 48 hours. In patients with renal insufficiency (baseline creatinine ≥1.5 mg/dl) ARF was defined by a rise in serum creatinine of ≥1 mg/dl from baseline over a period of 48 hours. Patients with elevated serum creatinine ≥1.5 mg/dl at discharge were categorized to have persistent renal insufficiency. All patients were treated on the intensive care unit (ICU) until platelet levels rose to more than 50 000/µl. Symptomatic treatment consisted of blood pressure control, electrolyte and water balance control, and whole blood transfusions if necessary.

“Remission” was defined as normalization of serum creatinine ≤1.2 mg/dl and reversal of neurological symptoms. All patients categorized as remission did not exhibit proteinuria at the time of discharge. Systolic blood pressure was normalized in 9 of 11 patients with renal insufficiency on admission and remission at discharge. Diastolic blood pressure was normalized in all these patients.

### Statistical Analysis

The objective of this study was (1) to analyse potential differences between patients with renal impairment and patients with normal renal function on admission, (2) to find potential risk factors for persistent renal insufficiency and (3) to find potential risk factors for mortality. For this purpose we used the non-parametric Mann-Whitney test and performed pairwise comparisons for the baseline factors CRP, blood pressure, platelets, LDH and white blood cell count (WBC). Additionally, SAP and MAP were defined with 140 and 100 mmHg as cut-off, and odds ratios (OR) and their 95% confidence intervals (CI) were assessed to describe the strength of association between these factors and the renal status on admission (situation 1).

For persistent renal insufficiency, the prognostic impacts of the baseline factors were first explored one at a time by logistic regression analyses, adjusted for renal status on admission. Factors associated with a p value of the Wald type <20% were examined more closely in a multivariate logistic regression model, using forward selection. Results are expressed as OR with their 95% CI. The variables CRP, WBC, platelets and LDH were natural logarithm transformed for inclusion in regression analyses (situation 2).

In situation 3, we analysed additionally to the parameters from situation 1 and 2 the factors age, haemoglobin, schistocytes and creatinine. Due to small sample sizes, a logistic regression analysis was not feasible, thus we used a non-parametric Mann Whitney test and performed pairwise comparisons for surviving and deceased patients.

If not stated otherwise, continuous variables were presented as median (interquartile range (IQR)), categorical variables were presented as proportions (%). Because of the explorative character of this study we did not adjust the significance level α = 0.05 to account for multiple testing. Therefore, all p-values are of an explorative nature and p values<0.05 were considered to be statistically significant. All reported p-values are two-sided. The analyses were performed using PASW Statistics 18.0.3 for Windows (SPSS 2010, Chicago, Il., USA).

## Results

### Clinical characteristics of patients on initial presentation

62 consecutive patients diagnosed with adult TMA were analysed in this study (table 1). Median age at presentation was 35 years with a wide range of 16 to 76 years (interquartile range (IQR): 27–49). Two thirds of our patients were female. 82% of patients only had a single episode of TMA whereas 18% relapsed at least once during the study period. Half of our patients exhibited neurological impairment varying from less severe symptoms such as headache and dizziness to severe seizures and coma. Renal insufficiency at presentation was very common (table 1). Most of our patients had no history of renal insufficiency prior to their first TMA episode. In patients with history of chronic renal failure, 3 patients had received a renal transplant, 2 patients had SLE, and one patient had scleroderma.

**Table 1:** Clinical characteristics of patients on admission.

	*n* (%)	Median (IQR)	Associated risk factors for the development of TMA	*n* (%)
Total number of patients	62		Infection	18 (29.0)
Age at first event (yr)		35 (27–49)	Pulmonary infection	5 (8.1)
Female gender	40 (64.5)		Diarrhea	7 (11.3)
Male gender	22 (35.5)		Pregnancy / oral contraceptives	8 (12.9)/2 (3.2)
Patients with single event	51 (82.3)		Renal transplantation	4 (6.5)
Patients with relapsing TMA	11 (17.7)		Malignancy	4 (6.5)
Neurological symptoms	32 (51.6)		SLE	3 (4.8)
Renal impairment	39 (62.9)		Systemic sclerosis	2 (3.2)
Dialysis treatment	32 (51.6)		Drugs	2 (3.2)
			Unknown	19 (30.6)

IQR: Interquartile range.

The different underlying causes of TMA in our patients are summarized in table 1. 31% of all patients had no obvious clinical trigger for the development of TMA.

19% of our patients were known to suffer from hypertension prior to the onset of TMA, whereas 81% did not show any medical history of hypertension.

### Clinical outcome

At discharge, remission (no renal insufficiency, no proteinuria, no neurological symptoms) was achieved in 42% of patients (table 2). Renal failure had resolved in 11 of 39 patients. The number of dialysis-dependent patients decreased from 52% to 23% (table 2). Only two patients, one with renal insufficiency on admission and one without, still had a neurological deficit at discharge. Among those patients with no previous hypertension, 32% required antihypertensive treatment at the time of discharge. 7 patients with TMA died (table 2), one of sepsis, three of severe cerebral hemorrhage, and three of TMA-associated acute myocardial infarction where immediate lysis therapy was unsuccessful.

**Table 2:** Clinical outcome.

	All patients*n* (%)	Renal impairment on admission*n* (%)	Normal renal function on admission (n = 23)*n* (%)
Remission	26 (41.9)	8 (20.5)	18 (78.3)
Renal insufficiency without dialysis	14 (22.6)	10 (25.6)	2 (8.7)
Dialysis	14 (22.6)	11 (28.2)	0 (0)
Neurological deficit	2 (3.2)	1 (2.6)	1 (4.3)
Death	7 (11.3)	5 (12.8)	2 (8.7)

### Clinical markers for renal insufficiency on admission

C-reactive protein (CRP) levels on admission were significantly higher in patients with renal insufficiency compared to patients with normal renal function (table 3, figure 1). Taking the median of CRP values (2.7 mg/dl) to divide patients into two subgroups, 10 patients with CRP≥2.7 mg/dl had infections whereas 20 patients did not have signs of infection (6 patients with unknown trigger of TMA, 5 patients post-partum, 3 patients with tumour, 3 patients with drug-induced TMA, 2 patients with SLE).

**Figure 1:** Risk factors for renal insufficiency in TMA. A: CRP serum levels on admission are significantly higher in patients with renal insufficiency compared to patients with normal renal function. B: Systolic arterial pressure (SAP) and mean arterial pressure (MAP) on admission are significantly higher in TMA patients with renal insufficiency.

**Table 3:** Characteristic factors for acute renal failure on admission.

	All patients (*n* = 62)Median (IQR)	Renal impairment (*n* = 39)Median (IQR)	Normal renal function (*n* = 23)Median (IQR)	p-value(Mann-Whitney-U test)
MAP (mmHg)	106 (90–117)	110 (95–120)	97 (87–110)	**0.027** *
SAP (mmHg)	140 (120–150)	150 (130–160)	130 (120–140)	**0.009** *
DAP (mmHg)	85 (70–100)	89 (80–100)	80 (70–90)	0.067
CRP (mg/dl)	2.7 (0.9–5.4)	2.9 (1.4–8.7)	0.95 (0.3–2.8)	**0.003** *
Platelets (/µl)	25 000 (9 000–56 000)	40 000 (18 000–85 000)	9 000 (8 000–26 000)	**0.001** *
LDH (U/l)	1 259 (714–2 001)	1 430 (765–2 799)	1 002 (630–1 650)	0.147
WBC (/µl)	10 800 (7 000–13 500)	11 900 (7 100–15 600)	9 400 (6 200–12 000)	0.062

*values significantly higher in patients with impaired renal function compared to patients with normal renal function on admission (p<0.05). IQR: Interquartile range.

Blood pressure levels, MAP and SAP, were also significantly higher in patients with renal impairment on admission (table 3, figure 1). Patients with SAP>140 mmHg on admission had a sevenfold increased probability of renal insufficiency on admission (odds ratio (OR) 7.464, CI 2.097–26.565). Patients with MAP>100 mmHg on admission had a fourfold increased probability (OR 4.261, CI 1.400–12.972) of acute renal insufficiency. There was a tendency for lower DAP in patients with normal renal function. Platelet count was significantly lower in patients with normal renal function (Table 3). This finding reflects the high proportion of patients with a clinical diagnosis of TTP in this group who often present with very low thrombocyte counts but with normal renal function. No significant difference was observed for LDH levels or white blood cell count (WBC), as described previously [21].

In our study, schistocytes remained elevated in some patients although LDH levels and platelet count were already normalized (data not shown). Therefore, as published earlier [22], schistocytes were unreliable markers for the detection of disease activity.

### Risk factors for persistent renal insufficiency

Our objective of this study was to identify clinical markers to detect patients at risk for TMA-induced sustained renal insufficiency. We performed logistic regression analyses, adjusted for renal status on admission (table 4), comparing patients on admission and at discharge. Potential risk factors influencing renal status at discharge were high MAP, SAP, DAP, and LDH levels on admission (table 4). We observed a strong association of elevated MAP on admission with renal insufficiency at discharge in multivariate analysis (table 5). An increase in MAP by 10 mmHg was associated with a twofold increased chance for renal insufficiency at discharge. This finding indicates that patients with renal dysfunction on admission as well as at discharge have higher blood pressure levels compared to patients with normal renal function.

**Table 4:** Risk factors for renal insufficiency at discharge. Logistic regression analyses, adjusted for renal status on admission.

	Renal impairment on admission only (*n* = 8)Median (IQR)	Renal impairment on admission and at discharge (*n* = 26)Median (IQR)	Normal renal function on admission and at discharge (*n* = 19)Median (IQR)	p-value(Wald-Test)
MAP (mmHg)	96 (88–111)	113 (105–124)	93 (83–107)	**0.011** *
SAP (mmHg)	133 (120–148)	150 (139–173)	120 (110–140)	**0.025** *
DAP (mmHg)	80 (70–93)	90 (80–100)	80 (70–90)	**0.023** *
CRP (mg/dl)	2.75 (1.1–4.9)	2.9 (1.5–9.5)	1.1 (0.3–3.9)	0.816
LDH (U/l)	1 835 (1 038–3 655)	1 346 (670–2 001)	1 002 (630–1 650)	**0.082** *
WBC (/µl)	11 900 (6 600–13 900)	11 050 (7 000–16 300)	9 400 (6 100–12 000)	0.894

*values higher in patients with impaired renal function compared to patients with normal renal function at discharge (p<0.20). IQR: Interquartile range.

**Table 5:** Risk factors for renal insufficiency at discharge, multivariate logistic regression analysis.

	*β* (a)	SE(b)	p-value (Wald Test)	Odds Ratio (95% CI)
Renal impairment on admission(c)	3.290	0.927	<0.001	26.84 (4.36–165.11)
MAP (mmHg)	0.070	0.028	0.011	1.07 (1.02–1.13)
Constant	−12.869	3.630	<0.001	

(a) *β*, estimated regression coefficient,

(b) standard error of *β*,

(c) “yes” coded 1.

In our logistic regression analysis (table 4), LDH levels were higher in patients with renal impairment on admission and at discharge compared to patients with normal renal function.

### Risk factors for death from TMA

The only associated risk factor for death in our study population was older age (table 6). MAP, SAP, DAP, LDH levels, CRP levels, WBC, haemoglobin levels, thrombocyte counts, schistocyte levels or creatinine levels were not significantly different in patients who died from TMA compared to surviving patients. Multivariate analysis was not performed due to the small number of deceased patients.

**Table 6:** Risk factors for TMA-associated death.

	Surviving patients(*n* = 55)Median (IQR)	Deceased patients(*n* = 7)Median (IQR)	p-value
Age (yrs)	34 (26–45)	48 (41–65)	0.009 *
MAP (mmHg)	106 (93.33–116.67)	95 (90–106.67)	0.346
SAP (mmHg)	140 (120–150)	130 (120–150)	0.512
DAP (mmHg)	87 (70–100)	80 (70–85)	0.280
LDH (U/l)	1 241 (694–1 935)	1 430 (1 086–3 570)	0.171
CRP (mg/dl)	2.5 (0.9–4.4)	3.6 (2.2–8.7)	0.386
WBC (/µl)	10 600 (6 400–13 800)	12 600 (10 000–13 500)	0.182
Hemoglobin (g/dl)	8.2 (7.1–9.8)	7.7 (5.7–11.3)	0.730
Platelets (/µl)	26 000 (9 000–58 000)	12 000 (5 000–56 000)	0.344
Schistocytes per field of view	6 (3–9)	7 (7–8)	0.528
Creatinine (mg/dl)	2.5 (1–5.2)	1.5 (1–4.3)	0.815

IQR: Interquartile range.

## Discussion

TMA is a life-threatening disease that was previously associated with a high mortality of more than 90% before plasmapheresis was introduced as therapy for TMA patients. Nowadays, survival rates have significantly improved, but sporadic non-Shiga-toxin-induced HUS still has a mortality rate of up to 50% in some patient subgroups [17]. The 2011 outbreak of *E.coli O104:H4* in Germany demonstrated the severity of this disease very clearly, where at least 27 patients died from diarrhea-associated HUS [6].

This study was designed to evaluate clinical risk factors predisposing TMA patients to renal insufficiency. The clinical course of a single patient presenting with TMA is often difficult to predict. Therefore, we analyzed data of 62 consecutively treated TMA patients to identify markers for the development of renal insufficiency and for the lack of renal recovery after successful TMA treatment.

Attempts to clinically define prognostic factors for the development of renal insufficiency in TMA have already been made earlier [21], [23], [24], [25]. Hollenbeck and co-workers demonstrated the importance of plasmapheresis to prevent the development of end-stage renal disease compared to plasma infusion alone [21]. In three studies pre-existing nephropathy or severe renal involvement were identified as risk factors for chronic renal failure [23], [24], [25]. Four studies correlated chronic renal failure to the severity of arterial and glomerular damage on renal biopsy [23], [24], [25], whereas one study did not find any correlation between renal histology and renal prognosis [21]. Compared to the present analysis patient subgroups were different. In the study by Hollenbeck et al. only 71% of patients were treated with plasmapheresis. Tostivint and colleagues reported exclusively on HUS patients, not on TTP patients, mostly treated with plasma infusion [23], with a large cohort of HIV positive cases. In our study patients were treated almost exclusively with plasmapheresis.

Acute renal failure (ARF) in TMA patients is frequently seen. In our study, more than 60% of patients showed renal impairment at presentation confirming results that have been published earlier (for review, see [17],[26],[27]). We identified high CRP and high blood pressure as clinical markers associated with ARF in TMA patients. CRP serum levels on admission were significantly increased in patients with ARF compared to patients with normal renal function. Therefore, high CRP may serve as a risk factor for ARF in TMA. CRP is a non-specific acute phase protein synthesized and degraded in the liver. It is markedly elevated in septic states in which ARF develops with a prevalence of 9–40% [28]. In our study, sepsis only played a minor role as a potential cause of ARF. The reason for high CRP levels in our patient subgroup with ARF is unclear. They usually occur in response to infection and inflammation. In the renal insufficiency group they may reflect additional, clinically undetected infection, possibly facilitating the development of ARF. Since WBC was not elevated in patients with higher CRP levels it is unlikely that severe infections were the reason for CRP elevation. Therefore, high CRP levels should rather be interpreted as an indicator for the severity of TMA-induced organ damage, including the kidney. Going along the same line with our observation, a Japanese study on diarrhea-associated typical HUS in children (D+ HUS) identified high CRP serum levels as a risk factor for the development of severe CNS disorders [29]. High CRP has also been recognized as a prognostic indicator in chronic renal disease. [30], [31]. Serum CRP levels predict death in dialysis patients [32], [33]. In severe renal insufficiency, elevation of CRP is associated with a higher cardiovascular mortality due to the contribution of CRP in endothelial damage and atherogenesis [34], [35]. CRP might therefore play an active role in endothelial damage also in TMA patients, independently of its elevation in septic states. Thus, high CRP levels may reflect TMA activity itself, leading to more severe end-organ damage and ARF.

In our cohort, high blood pressure (MAP) in patients with renal insufficiency on admission was a risk factor for acute and persistent renal insufficiency. Tostivint and co-workers already indicated that high DAP was associated with chronic renal failure but they did not identify high DAP as independent risk factor in multivariate analysis [23]. Higher blood pressure is either due to pre-existing hypertension or due to secondary hypertension caused by TMA-related renal involvement. Interestingly, only a minority of patients was known to be hypertensive prior to their episode of TMA. Most of our patients also did not have any previous history of kidney disease. Our data suggest that adequate treatment of hypertension in TMA patients may be essential to prevent additional renal damage. By lowering blood pressure into the normal range renal function might be preserved and may lead to a better renal outcome.

LDH serum levels at the time of admission were higher in patients with sustained renal insufficiency at discharge compared to patients with normal renal function. This finding is not surprising since LDH levels indicate the severity of hemolysis and of end-organ damage. Higher LDH levels in patients with persisting renal insufficiency suggest a more severe course of TMA and presumably also more severe kidney damage.

Several risk factors for the development of TMA, such as infection, pregnancy, autoimmune disease or drugs, have been published. We found these to be present in 69% of our patients. One third of patients did not show any apparent trigger. Genetic testing of genes encoding complement factors and determination of ADAMTS13 activity have been demonstrated to be useful to clarify the etiology of TMA [12]. Recent studies show that 20% of HUS patients have a familiar form of HUS [26], and 80% of TTP is triggered by deficient activity of ADAMTS13 [12]. Unfortunately, these data were only available in a minority of our patients.

11% of patients in our study died due to sepsis, hemorrhage, and acute myocardial infarction. This mortality rate is comparable to mortality rates previously published for this disorder [17], [25], [36]. We identified older age as a risk factor for death confirming results of Shiepatti and co-workers [24]. We did not observe any association between risk of death and blood pressure, CRP serum levels, LDH serum levels, Hb, WBC, thrombocytes, schistocytes, or creatinine serum levels on admission. Data published earlier suggested that low hemoglobin levels as well as high WBC were also associated with a higher risk of death [21]. In our study, we were not able to confirm these findings. This may reflect differences between patient subgroups in both studies.

For interpretation of this study some limitations should be taken into account. The study took place in a single hospital with a particular clientele of patients that might be different compared to hospitals in other regions or other countries. For example, we did not observe any HIV infections in our patient cohort. Furthermore, a single site investigation often presents data on only a limited number of cases.

In summary, we were able to identify parameters significantly correlated with unfavorable outcomes in TMA patients. High CRP serum levels and high blood pressure indicate a predisposition for ARF and persistent renal insufficiency. These parameters could help to detect TMA patients at risk for sustained kidney function impairment. Therapy of the underlying cause of CRP elevation as well as immediate and sufficient lowering of blood pressure may improve renal prognosis.
